# Effects of Recombinant Human Epidermal Growth Factor Eye Drops Combined with Phacoemulsification on Short- and Long-Term Visual Acuity Recovery and Related Dry Eye Complications in Patients with Senile Cataract

**DOI:** 10.1155/2022/1041558

**Published:** 2022-06-28

**Authors:** Lingzhi Fan, Tao He, Jiguang Shi, Xianlin Ke, Xiaolei Lu

**Affiliations:** ^1^Glaucoma and Cataract Department, Enshi Huiyi Ophthalmic Hospital, Enshi, Hubei 445000, China; ^2^Ophthalmologic Center, Hubei General Hospital, Wuhan, Hubei 430061, China

## Abstract

**Objective:**

To investigate the effects of recombinant human epidermal growth factor eye drops combined with phacoemulsification on short- and long-term visual acuity recovery and related dry eye complications in patients with senile cataract.

**Methods:**

Sixty patients with senile cataract cured from January 2019 to January 2021 were enrolled in our hospital. The patients in the control group were arbitrarily assigned into the control and the research group. The former group received phacoemulsification, and the latter group received recombinant human epidermal growth factor (RhEGF) eye drops combined with phacoemulsification. The curative effect, the incidence of xerophthalmia, short-term and long-term vision improvement, changes of corneal endothelial cells, serum factors, and life quality scores were compared.

**Results:**

The effective rate of the research group was 90.00%, and the effective rate of the control group was 66.67%; the curative effect of the research group was higher than that of the control group (*P* < 0.05). The incidence of dry eye in the research group was lower than that in the control group (*P* < 0.05). The short-term and long-term visual acuity improvement effect of the research group was better than that of the control group (*P* < 0.05). After treatment, the density of corneal endothelial cells in the research group was higher than that in the control group, while the proportion of hexagonal cells and the coefficient of variation of corneal endothelial cells in the research group were lower than those in the control group (*P* < 0.05). After treatment, IL-6 and TNF-*α* in the research group were lower than those in the control group (*P* < 0.05). Compared with the control group, the physical function, psychological function, social function, and healthy self-cognition scores of the research group were all lower (*P* < 0.05).

**Conclusion:**

Cataract is the leading cause of blindness in the world. With the continuous improvement of cataract phacoemulsification technology, the incidence of some serious complications has gradually lessened. Xerophthalmia is one of the most obvious and predictable complications after cataract surgery and may affect the recovery of postoperative visual acuity. Recombinant human epidermal growth factor eye drops can effectively enhance the visual acuity of patients, promote the curative effect, and strengthen the life quality.

## 1. Introduction

Cataract is one of the global eye diseases that cause blindness [1]. With the continuous enhancement of medical technology, cataract surgery has changed from vision surgery to intraocular refractive surgery and to minimally invasive, individualized, and accurate. Although phacoemulsification with intraocular lens implantation is a popular surgical method at present, there are still various complications [1, 2]. In the early stage after phacoemulsification, some patients will have symptoms such as corneal edema and poor vision recovery, and irreversible loss of corneal endothelial cells and cystoid macular edema may occur with the passage of time. It is related to the surgeon's proficiency, the mode of operation, the hardness of the nucleus, and the phacoemulsification instrument adopted [2].

Since the 1980s, phacoemulsification has been vigorously carried out in clinic with less injury, quick recovery, and good benefit [3]. While the operation brought light to people, some patients with preoperative xerophthalmia aggravated postoperative xerophthalmia, and some patients without preoperative xerophthalmia developed symptoms such as dry eyes, foreign body sensation, and even blurred vision after operation, accompanied by shortened tear film rupture time (BUT), corneal fluorescent staining, reduced basal tear secretion, meibomian gland dysfunction, and destruction of ocular surface tissue [3]. This leads to the symptoms of eye discomfort and greatly reduces the life quality of patients. The problem of postoperative xerophthalmia has been widely concerned by ophthalmologists. It has important clinical significance and great clinical prospect for the prevention and treatment of xerophthalmia after phacoemulsification. In 2002, Liu et al. reported that there were remarkable changes in tear film after phacoemulsification and Wu Na reported in 2012 that BUT in diabetes with cataract group within 1 month after operation was remarkably lower compared to before operation, tear film gradually recovered 3 months after operation, and BUT gradually approached the preoperative level, while there was no remarkable change in BUT in simple cataract group before and after operation [3, 4]. BUT in diabetes with cataract group at 3 months after operation was remarkably shorter compared to simple cataract group. The tear secretion test and corneal fluorescent staining indicated similar results. The BUT recovery time of diabetic patients with cataract after phacoemulsification was longer compared to cataract patients without cataract. Diabetic patients with cataract after cataract surgery are more likely to have dry eyes, and the recovery of tear film stability is more difficult and longer.

Phacoemulsification is relatively simple and effective, but the operation is a traumatic operation, which will bring damage to patients and cause postoperative complications [4]. Xerophthalmia is a common complication after cataract phacoemulsification, which will affect the improvement of patients' vision and recovery of the disease, so it is necessary to take scientific methods to treat xerophthalmia after phacoemulsification. At present, eye drops are generally adopted to interfere with postoperative xerophthalmia [5]. Recombinant human epidermal growth factor (RhEGF) is a kind of cell growth factor composed of many kinds of amino acids, and RhEGF eye drops can effectively promote cell division and receptor binding to a certain extent, activate cells, cause cell cascade reaction, increase protein, RNA, and DNA synthesis, accelerate cell metabolism, promote the proliferation of corneal epidermal cells, and accelerate the proliferation and differentiation of corneal epithelial stem cells [6]. In addition, it can stimulate the proliferation of fibrous cells and corneal stroma and enhance the arrangement of collagen lamella [6, 7]. Optogenetics is a technique that combines optics and genetics to control specific neurons, which is widely applied in the peripheral nervous system, such as vision study [7]. The use of this drug after phacoemulsification can accelerate the regression of symptoms, shorten the recovery time of patients, and repair corneal endothelial cells and corneal injury [8]. Based on this, this study focuses on the effects of recombinant human epidermal growth factor eye drops combined with cataract phacoemulsification on short- and long-term visual acuity recovery and related dry eye complications in patients with senile cataract.

## 2. Patients and Methods

### 2.1. General Information

Sixty patients with senile cataract cured from January 2019 to January 2021 were enrolled in our hospital. The patients were arbitrarily assigned into control and research group. In the former group, the age was 61-86 years old, with an average of 71.44 ± 3.53 years, including 18 males and 12 females, while in the latter group, the age was 44-76 years old, with an average of 71.57 ± 3.56 years, including 16 males and 14 females. There exhibited no statistical significance in the general data. This study was permitted by the Medical Ethics Association of our hospital, and all patients noticed informed consent.

Inclusion criteria: (1) all patients of dry eye were diagnosed by visual acuity, slit lamp, and ultrasonic examination [9]; (2) all patients underwent phacoemulsification, and there was no surgical taboo.

Exclusion criteria: (1) complicated with eyelid insufficiency, lacrimal duct disease, keratoconjunctivitis, pterygium, and other eye diseases; (2) complicated with eyelid insufficiency, lacrimal duct disease, keratoconjunctivitis, pterygium, and other eye diseases; (3) he has a history of eye surgery in the past 3 months and has used drugs that affect tear secretion in the past month; (4) exclusion of patients with congenital nonlacrimal disease and no lacrimal gland.

### 2.2. Treatment Methods

The control group received phacoemulsification: preoperative preparation: laboratory examination, slit lamp microscope examination, intraocular pressure (Topcon noncontact tonometer), intraocular lens biological measurement (AL-Scan optical biometric instrument), uncorrected and corrected visual acuity (Topcon computer optometry), corneal endothelioscopy (SP-2000P keratometer), B-ultrasound (QuentelMedical AB ultrasound), ECG, chest positive film, and OCT fundus examination (SD-OCT, Heidelberg, Germany). Parameter setting: test group (main control fluid flow system) intraoperative fluid flow rate 30 cc/min, negative pressure 525 mmHg, IOP 55 mmHg, twist energy 60%; control group (gravity flow system) high 95 cm, liquid velocity 40 cc/min, torsion energy 60%, and negative pressure 500 mmHg. All patients were treated with 0.5% levofloxacin eye drops (clonbital) 4 times a day for 3 consecutive days.

The surgical procedures were performed by Centurion phacoemulsification instrument and ZeissS88 operating microscope, operated by the same skilled doctor. Operation procedure: 0.4% obucaine (Benoxil) topical anesthesia, patient lying flat, routine disinfection field skin, Baotou, hole towel, paste aseptic eye patch, eyelid opener to open face, rinse conjunctival sac with 0.5% povidone iodine, after 30 seconds, and rinse clean with 3 : 2 sterile eyes with a mixture of balanced salt solution and tobramycin injection. 3 mm transparent corneal incision was performed in the limbus at about 10 : 00-11 : 00, corneal endothelium and anterior chamber were protected with viscoelastic, continuous circular capsularhexis, about 5.5~6 mm in diameter, lateral corneal incision at about 2 : 00, water separation, nucleus splitting, phacoemulsification, injection of cortex, posterior capsule polishing, injection of viscoelastic agent, implantation of intraocular lens into bag, absorption of viscoelastic with injection handle, and watertight incision with perfusion fluid. It is necessary to apply tobramycin dexamethasone eye ointment into the conjunctival capsule (Dian Bishu), a single blindfold.

Research team: on the basis of the control group, the patients were treated with RhEGF eye drops (specification: 40000 IU/4 ml/branch, trade name: Yibei, Chinese medicine standard: WS4- (S-061)-2005Z, and manufacturer: Guilin Huanowei Genome Pharmaceutical Co., Ltd.); two times a day, one drop per time, for 6 weeks.

### 2.3. Observation Indicators

#### 2.3.1. Curative Effect

Criteria for judging curative effect [10]: under the slit lamp, the corneal display is normal, the corneal fluorescence staining disappears or basically disappears, and the disappearance of ocular foreign body, dryness, photophobia, and other symptoms can be recorded as remarkable effect; under the slit lamp, the corneal fissure is not obviously normal, the corneal fluorescence staining disappears and improves, and the symptoms such as ocular foreign body, dryness, and photophobia can be recorded as effective; under slit lamp, no remarkable reduction of corneal fissure, disappearance of corneal fluorescence staining, no improvement of ocular foreign body, dryness, photophobia, and other symptoms can be recorded as invalid.

#### 2.3.2. Incidence of Dry Eye Syndrome

The incidence of xerophthalmia was calculated.

#### 2.3.3. Short-Term and Long-Term Vision Improvement

Patients were followed up for 3 months and 1 year, respectively, and the number of visual acuity improvement was counted.

#### 2.3.4. Changes of Corneal Endothelial Cells

The changes of corneal endothelial cells before and after treatment were analyzed. 100 to 150 cells in the central area of cornea were counted and examined by noncontact endothelioscope. Clear images were taken after taking pictures (3 times in a row). The proportion of hexagonal cells, the density of corneal endothelial cells, and the coefficient of variation of corneal endothelial cells were calculated.

#### 2.3.5. Serum Factor Detection

The patient's tears (15 *μ*l) were collected by capillary method, enzyme linked immunosorbent assay (ELISA) was adopted to detect tumor necrosis factor-*α* (tumor necrosis factor-*α*, TNF-*α*), and the level of interleukin-6 (IL-6) was detected.

#### 2.3.6. Life Quality Scale

The life quality scale consists of four subscales, including physical, psychological, social, and health self-awareness, with a total of 29 items [11]. The Cronbach's *α* coefficient of the scale is 0.79 to 0.91. The scale was scored by 1-5 grades. The lower the score, the higher the satisfaction.

### 2.4. Statistical Analysis

Using SPSS21.0 statistical software, before statistical analysis, the measurement data were examined by normal distribution and variance homogeneity analysis to meet the requirements of normal distribution or approximate normal distribution, presented as $\bar{x}\pm s$, and repeated measurement data were analyzed by repeated measurement analysis of variance. *T* test was adopted to compare the two groups, *n* (%) was employed as an example to represent the counting data, and *χ*^2^ test was adopted to show that the difference exhibited statistically remarkable (*P* < 0.05).

## 3. Results

### 3.1. Comparison of Curative Effects

The curative effect of the research group was remarkably effective in 22 cases, effective in 5 cases and ineffective in 3 cases, with an effective rate of 90.00%; In the control group, 12 cases were markedly effective, 8 cases were effective, and 10 cases were ineffective, and the effective rate was 66.67%. The curative effect of the research group was higher (*P* < 0.05). All the data results are indicated in Figure 1.

### 3.2. Comparison of the Incidence of Dry Eyes

The incidence of xerophthalmia in the research group 6.67% (2/30) was lower compared to the control group 23.33% (7/30) (*P* < 0.05).

### 3.3. Comparison of Short-Term and Long-Term Vision Improvement

With regard to the effect of short-term and long-term vision improvement, the short-term and long-term vision improvement effect of the research group was better (*P* < 0.05). All the data results are indicated in Figure 2.

### 3.4. Comparison of Changes of Corneal Endothelial Cells

There exhibited no remarkable difference in the repair of corneal endothelial cells before treatment (*P* > 0.05). After treatment, the density of corneal endothelial cells in the research group was higher, while the proportion of hexagonal cells and the coefficient of variation of corneal endothelial cells in the research group were lower (*P* < 0.05). All the data results are indicated in Table 1.

### 3.5. Comparison of Serum Factors

There exhibited no remarkable difference in serum factors before treatment (*P* > 0.05); after treatment, the levels of IL-6 and TNF-*α* lessened, and the levels of IL-6 and TNF-*α* in the research group were lower (*P* < 0.05). All the data results are indicated in Table 2.

### 3.6. Comparison of Life Quality Scores

There exhibited no remarkable difference in the score of life quality before treatment (*P* > 0.05). After treatment, the score of life quality lessened. Compared between the two groups, the scores of physiological function, psychological function, social function, and health self-cognition in the research group were lower (*P* < 0.05). All the data results are indicated in Table 3.

## 4. Discussion

Visual impairment caused by cataracts afflicts tens of millions of people around the world and is the leading cause of global blindness [12]. With the accelerated deepening of the aging of China's population, the prevalence of cataract continues to rise, while the number of elderly patients with severe cataract is also greatly augmented. At present, the main treatment of cataract is phacoemulsification with intraocular lens implantation. With the continuous updating and improvement of phacoemulsification equipment, whether for operators or patients, the efficiency and safety of cataract surgery have reached a higher level [13]. Every phacoemulsification platform should aim to provide an energy-saving, time-saving, and safe surgical system with a minimum incidence of complications [14]. At present, phacoemulsification, as the main means for the treatment of cataract, has a good effect, which can not only remarkably enhance the visual acuity of patients but also obtain ideal visual quality. However, surgery will inevitably be accompanied by related complications. Many complications are easy to occur during and after phacoemulsification, such as, intraoperative rupture of posterior capsule, corneal endothelial injury, posterior corneal elastic layer detachment, iris injury, sharp increase of intraocular pressure, postoperative corneal edema, macular edema, and retinal detachment [15]. The factors of complications come from many aspects: the mode of phacoemulsification, mechanical factors, continuous washing of perfusion fluid and the use of phacoemulsification instrument are all important factors affecting intraoperative and postoperative complications of phacoemulsification [16].

At present, it is believed that the mechanism of xerophthalmia after phacoemulsification combined with intraocular lens implantation is as follows: (1) excessive use of antibiotic eye drops and topical anesthetic and improper washing of povidone iodine solution will have toxic effects on corneal epithelium, affect the permeability of corneal epithelial cells, and cause corneal epithelial cell damage. The stability of tear film lessened, and the degree of corneal fluorescent staining augmented; (2) the surgical incision can cut off the nerve fibers of the limbal and block the nerve conduction, resulting in the decrease of local corneal sensitivity, the decrease of blink activity, and the shortening of BUT; (3) intraoperative mechanical injury of ocular surface tissue, intraoperative and postoperative inflammatory reaction, tissue edema, delayed wound healing, and local eminence of surgical incision can all affect the incompleteness of corneal epithelium. The loss of adhesion-related cytoskeleton structure in the mucin layer in tear film leads to the decrease of tear film stability and the expression of inflammatory cytokines, which can further lead to ocular surface injury and form a vicious circle; (4) the exposure time of ocular surface light during operation can also cause damage to ocular surface tissue. Artificial tears are the main treatment for all degrees of xerophthalmia. Artificial tears can increase tear film stability, reduce ocular surface pressure, reduce dry eye symptoms, improve visual contrast sensitivity and optical quality, and improve the life quality [16, 17]. Artificial tears whose main ingredient is sodium hyaluronate are commonly used in clinic. There is a lack of research data on whether preoperative use of artificial tears can prevent and treat xerophthalmia after phacoemulsification in cataract patients with or without xerophthalmia.

In the consensus of dry eye clinical diagnosis and treatment experts issued in 2013 by the keratology group of Chinese Medical Ophthalmology Association, dry eye is defined as tear film instability and/or ocular surface damage caused by abnormal quality or quantity or hydrodynamics of tears [17]. This leads to symptoms of eye discomfort and visual dysfunction. The symptoms of xerophthalmia are dryness, foreign body sensation, burning sensation, easy fatigue, fear of light and wind, etc., which affect the life quality of patients and have become a serious public health problem in recent years. The existing epidemiology in China shows that the incidence of dry eyes in China is 21% to 30%. The risk factors are aging, women, high altitude, diabetes, pterygium, use of video terminals, abuse of eye drops, air pollution, corneal refractive surgery, allergic diseases, and some systemic diseases [18]. The Tear Film & Ocular Surface Society (TFOS) held its second meeting (TFOS DEWS II) in March 2015 and identified tear hyperosmosis as the core mechanism leading to dry eyes [19]. On the one hand, hypertonic tears promote the formation of inflammation; on the other hand, accelerate the apoptosis of corneal and conjunctival epithelial cells and goblet cells, and further aggravate the instability of tear film. Inflammation caused by tear film instability and hyperosmosis also leads to neurogenic chronic inflammation, which increases the severity of the disease and leads to a vicious circle [20]. In addition, many studies have indicated that the occurrence of xerophthalmia is closely related to the apoptosis of corneal epithelial cells, lacrimal gland cells, corneal endothelial cells, and conjunctival epithelial cells [21–23]. Abnormal apoptosis of ocular surface cells and suppressed apoptosis of lymphocytes in local ocular surface tissues eventually aggravate the inflammatory response [24]. At present, the treatment of dry eyes includes drug treatment and nondrug treatment, including artificial tears, promotion of tear secretion, anti-inflammatory drugs, surgery, diet adjustment, environmental factors, and supplementary therapy. Artificial tear replacement therapy is the main treatment for dry eyes. The types of artificial tears include viscosity enhancers, osmotic protective agents, and serum products [25]. Ideal artificial tear, its osmotic pressure, ion composition, and pH are the same or similar to those of tears, and it also contains simulated mucin and is close to tear viscosity [26]. Sodium hyaluronate is adopted as a viscosity enhancer by increasing the thickness of tear film, preventing dryness, promoting tear retention and protecting eye surface. It is widely adopted in clinic and can effectively simulate the function of secretory mucin. And then form an effective main structure of tear film, which plays a certain role in promoting the stable and effective combination of patients' epithelium and tear film [27]. RhEGF can increase the number of conjunctival goblet cells in patients with dry eyes, effectively promote the proliferation and division of tear film and corneal epithelial structure, reduce corneal epithelial damage, promote the change of tear film quality, and strengthen dry eye symptoms. Recombinant bovine basic fibroblast growth factor (r-bFGF) was adopted to treat xerophthalmia patients within one month after phacoemulsification, which could promote basic tear secretion, subjective dry eye sensation score, and corneal fluorescence staining score [28, 29]. Autologous serum contains the same growth factors as those in patients' tears, and the serum also contains anti-infective substances such as IgG, complement, and lysozyme, which can not only enhance the stability of tears but also promote the score of tiger red staining and ocular surface fluorescein staining and alleviate ocular inflammation. In addition, more attention has been paid to the damage of preservatives to the ocular surface. Even at very low doses, benzalkonium bromide, the most commonly used eye preservative, can cause inflammation in corneal epithelial cells, using artificial tears without preservatives. At present, there are few reports on the combination of sodium hyaluronate and rEGF without preservatives, and the therapeutic effect of the combination of sodium hyaluronate and rEGF in the elderly population with dry eyes is rarely reported [30–32].

In terms of the curative effect, the research group was remarkably effective in 22 cases, effective in 5 cases, and ineffective in 3 cases, with an effective rate of 90.00%; In the control group, 12 cases were markedly effective, 8 cases were effective, and 10 cases were ineffective; the effective rate was 66.67%. The curative effect of the research group was higher (*P* < 0.05). The incidence of xerophthalmia in the research group 6.67% (2/30) was lower compared to the control group 23.33% (7/30) (*P* < 0.05). With regard to the effect of short-term and long-term vision improvement, the short-term and long-term vision improvement effect of the research group was better (*P* < 0.05). There exhibited no remarkable difference in the repair of corneal endothelial cells before treatment (*P* > 0.05); after treatment, the density of corneal endothelial cells in the research group was higher, while the proportion of hexagonal cells and the coefficient of variation of corneal endothelial cells in the research group were lower (*P* < 0.05). There exhibited no remarkable difference in serum factors before treatment (*P* > 0.05); after treatment, the IL-6 and TNF-*α* lessened. Compared with the control group, the IL-6 and TNF-*α* of the research group were lower (*P* < 0.05). There exhibited no remarkable difference in the score of life quality before treatment (*P* > 0.05); after treatment, the score of life quality lessened. Compared between the two groups, the scores of physiological function, psychological function, social function, and health self-cognition in the research group were lower (*P* < 0.05). The analysis shows that the occurrence of xerophthalmia is closely related to the apoptosis of corneal epithelial cells, lacrimal gland cells, corneal endothelial cells, and conjunctival epithelial cells. In the meantime, abnormal apoptosis of ocular surface cells and suppressed apoptosis of lymphocytes in local ocular surface tissues eventually aggravate the inflammatory response [33–35]. The two can influence each other. Recombinant epidermal growth factor has been proved to promote the division and proliferation of corneal and conjunctival epithelium, promote the repair of ocular surface injury, maintain normal corneal epithelial structure, promote the change of tear film quality, reduce dry eye symptoms, and promote the change of tear film quality. The results of Hao Lili et al. indicated that the concentration of TGF*β*2 in tears in Sjogren's syndrome group and non-Sjogren's syndrome group was remarkably higher compared to normal control group [36–38]. Abnormal expression of TGF-*β*1 and augmented apoptosis of epithelial cells are closely related to type 2 diabetes mellitus complicated with xerophthalmia. Recombinant bovine basic fibroblast growth factor (r-bFGF) was adopted to treat xerophthalmia patients within one month after phacoemulsification, which could promote basic tear secretion, subjective dry eye sensation score, and corneal fluorescence staining score, indicating that this method is effective when treating xerophthalmia after phacoemulsification [39]. The results of Chen Yanya's study indicated that the expression rate of TGF*β*1 in conjunctival epithelial cells was different in patients with different degrees of dry eyes and positively correlated with conjunctival Lisamine green staining score, corneal fluorescein sodium staining score, and dry eye questionnaire score, and negatively correlated with TBUT and tear secretion test, that is, the higher the expression of TGF*β*1, the higher the degree of xerophthalmia [40–43]. Therefore, the therapeutic effect of sodium hyaluronate combined with RhEGF eye drops on xerophthalmia can also be achieved by reducing the rate of apoptotic cells and the secretion of TGF*β*1 and TGF*β*2 in the membrane of patients. Corticosteroids and nonsteroidal anti-inflammatory drugs (NSAIDs) can play an anti-inflammatory role by inhibiting the production of inflammatory mediators such as prostaglandins [44]. There are some limitations in this study. First, the sample size of this study is not large, and it is a single-center study, so bias is inevitable. In future research, we will carry out multicenter, large-sample prospective studies, or more valuable conclusions can be drawn.

Conclusively, cataract is the first cause of blindness in the world. With the continuous improvement of cataract phacoemulsification technology, the incidence of some serious complications has gradually lessened. Xerophthalmia is one of the most obvious and predictable complications after cataract surgery and may affect the recovery of postoperative visual acuity. Recombinant human epidermal growth factor eye drops can effectively enhance the visual acuity of patients, promote the curative effect, and strengthen the life quality.

## Figures and Tables

**Figure 1:** Comparison of curative effects between two groups.

**Figure 2:** Comparison of short-term and long-term vision improvement between two groups.

**Table 1:** Comparison of changes of corneal endothelial cells [$\bar{x}\pm s$].

Group	*N*	Corneal endothelial cell density (%)		Proportion of hexagonal cells		Coefficient of variation of corneal endothelial cells (unit/mm^2^)	
		Before treatment	After treatment	Before treatment	After treatment	Before treatment	After treatment
Control group	30	2005.38 ± 246.49	2235.91 ± 243.67	29.49 ± 6.45	34.94 ± 6.55	36.49 ± 7.34	34.29 ± 3.42
Research group	30	2006.49 ± 243.55	2634.92 ± 232.56	29.39 ± 6.77	43.29 ± 7.45	36.43 ± 7.53	29.19 ± 3.35
*t*		0.017	6.488	0.058	4.684	0.031	5.834
*P*		>0.05	<0.01	>0.05	<0.01	>0.05	<0.01

**Table 2:** Comparison of IL-6 and TNF- *α* ($\bar{x}\pm s$, pg/ml).

Group	*N*	IL-6		TNF-*α*	
		Before treatment	After treatment	Before treatment	After treatment
Control group	30	1426.94 ± 84.29	1294.44 ± 35.33	255.69 ± 12.43	222.59 ± 17.33
Research group	30	1428.77 ± 83.56	1102.56 ± 34.22	256.49 ± 12.34	192.84 ± 13.66
*t*		0.084	21.367	0.250	7.384
*P*		>0.05	<0.01	>0.05	<0.01

**Table 3:** Comparison of life quality scores before treatment ($\bar{x}\pm s$, points).

Group	*N*	Physiological function		Psychological function		Social function		Healthy self-cognition	
		Before treatment	After treatment	Before treatment	After treatment	Before treatment	After treatment	Before treatment	After treatment
Control group	30	15.78 ± 4.67	13.89 ± 2.46^a^	16.57 ± 3.55	14.66 ± 4.99^a^	18.31 ± 3.95	16.55 ± 2.34^a^	15.34 ± 3.64	13.86 ± 1.55^a^
Research group	30	15.76 ± 4.79	11.55 ± 2.54^b^	16.56 ± 3.83	12.12 ± 1.22^b^	18.84 ± 3.55	12.13 ± 3.31^b^	15.66 ± 3.61	10.83 ± 2.91^b^
*t*		0.016	3.624	0.010	2.708	0.564	5.972	0.341	5.033
*P*		>0.05	<0.01	>0.05	<0.01	>0.05	<0.01	>0.05	<0.01

## Data Availability

No data were used to support this study.
